This article has been retracted.

# Application Analysis of Multiacupoint Stimulation in Multimodal Labor Analgesia during the Whole Stage of Labor in Primipara

**DOI:** 10.1155/2022/5161562

**Published:** 2022-06-07

**Authors:** Lan Liu, Xin Men, Xiaohong Song, Xiaoxiao Qiu, Zhenzhao Huang, Jingyu Zhang, Hongda Yi, Pei Chen

**Affiliations:** ^1^Department of Anesthesiology, The Second Affiliated Hospital of Zhejiang University School of Medicine, Hangzhou, Zhejiang 310009, China; ^2^Department of Anesthesiology, Hangzhou Women's Hospital, Hangzhou, Zhejiang 310008, China; ^3^Department of Gynaecology, Hangzhou Women's Hospital, Hangzhou, Zhejiang 310008, China

## Abstract

**Purpose:**

To analyze the application value of multimodal analgesia (MMA) regimen of patient-controlled epidural analgesia (PCEA) combined with multiacupoint stimulation analgesia during the whole stage of labor analgesia in primipara.

**Methods:**

300 primiparas with natural delivery were selected. According to the different ways of labor analgesia, they were divided into the first stage of labor active period PCEA group (group A), the whole stage of labor PCEA group (group W), and the whole stage of labor PCEA combined with multiacupoint stimulation analgesia group (group WM). The effect of MMA during the whole-labor process on maternal and infant safety was evaluated. The specific observation indicators were as follows: visual analogue scale (VAS) scores before analgesia (*T*_0_), at full opening of the uterus (*T*_1_), at the end of the second stage of labor (*T*_2_), and at the end of the third stage of labor (*T*_3_); stress response indicators at *T*_0_ and *T*_1_: epinephrine (*E*), norepinephrine (NE), glucose (Glu), and *β*-endorphin (*β*-EP) levels; delivery time of each stage of labor; the Apgar score of newborns at 1 and 5 min after birth; indicators of umbilical artery blood gas analysis immediately after delivery: PH value, base excess (BE), partial pressure of oxygen (PaO_2_), and partial pressure of carbon dioxide (PaCO_2_); incidence of postpartum depression (PPD) at 6 weeks after delivery.

**Results:**

At *T*_1_, *T*_2_, and *T*_3_, the VAS scores were lower in groups W and WM than in group A, and the VAS scores were lower in group WM than in group W (*P* < 0.05). At *T*_0_, there was no significant difference in the comparison of *E*, NE, Glu, and *β*-EP levels among the three groups (*P* > 0.05). At *T*_1_, the levels of *E*, NE, Glu, and *β*-EP were higher in the three groups than in the same group at *T*_0_, the levels of *E*, NE, and Glu were lower, the levels of *β*-EP were higher in groups W and WM than in group A, and the levels of *β*-EP were higher in group WM than in group W (*P* < 0.05). Comparing the delivery time of the first stage of labor in the three groups, groups A and WM were shorter than group W (*P* < 0.05). Comparing the delivery time of the second and third stages of labor in the three groups, there was no significant difference (*P* > 0.05). Comparing the Apgar scores of the three groups of newborns at 1 and 5 min after birth, there was no significant difference (*P* > 0.05). Comparing the incidence of newborn asphyxia in the three groups, there was also no significant difference (*P* > 0.05). Comparing the PH, BE, PaO_2_, and PaCO_2_ of three groups of newborns after delivery, there were no significant differences (*P* > 0.05). At 6 weeks after delivery, the incidence of PPD was lower in groups W (10.00%) and WM (8.00%) than in group A (20.00%) (*P* < 0.05).

**Conclusion:**

The application of the MMA regimen of PCEA combined with multiacupoint stimulation for labor analgesia during the whole stage of labor in primipara can effectively reduce labor pain and stress response during the whole stage of labor and shorten the delivery time of the first stage of labor, the indicators of newborn Apgar score and umbilical artery blood gas analysis are not affected, and the incidence of PPD in patients is reduced, which can play a protective role for the safety of mother and infant.

## 1. Introduction

Childbirth is a physiological event, and the pain a woman experiences during childbirth is considered to be the most severe pain a woman experiences in her lifetime. It accompanies the whole delivery process of the puerperium, which not only triggers a series of neurological and endocrine reactions in the puerpera but also causes a strong psychological burden. The two influence and promote each other, thus forming a vicious circle, which will eventually lead to maternal consumption of a lot of physical strength to prolong the labor process and even cause fetal distress in the uterus, threatening the health of mothers and infants [1]. Based on this, some women choose cesarean section because of unbearable pain, but there are many complications after cesarean section, which can affect the postpartum recovery and physical health of the mother [2]. How to reduce the pain during childbirth, reduce the rate of cesarean section, ensure the smooth progress of natural childbirth, and improve the prognosis of obstetrics has become the key topic of current clinical research.

At present, the most commonly used and effective method of labor analgesia in clinical practice is intraspinal analgesia, which exerts an analgesic effect by blocking the conduction of nerve impulses [3], such as epidural block analgesia (CEA) and patient-controlled epidural analgesia (PCEA) [4]. Studies have found that epidural labor analgesia does not increase the rate of clinical cesarean section, but it is still difficult to comprehensively and accurately evaluate its impact on neonates [5, 6]. And epidural labor analgesia is mainly used in the active phase of the first stage of labor. It is still controversial whether the application of it in the first stage of labor, which has no obvious pain but is still accompanied by certain functional, metabolic, and psychological changes, will affect the progress of the labor process and delivery outcomes. In addition, nondrug and nontraumatic analgesia has been advocated internationally to increase the rate of natural childbirth, which is consistent with the view of traditional Chinese medicine in the motherland [7].

Acupoint analgesia has certain analgesic and hypnotic effects in clinical observation [8]. Common methods include acupuncture analgesia, auricular acupoint pressing, transcutaneous electrical nerve stimulation (TENS), acupoint injection, and acupoint massage. Domestic studies have found that applying TENS to labor analgesia, stimulating acupoints with specific frequency pulses to increase the body's pain threshold, can play a certain role in sedation and analgesia, but the results are poor when applied alone in the active period of the first stage of labor when pain is intense. In addition, the application of auricular acupoint pressing and acupoint injection during the whole stage of labor analgesia in primipara also has the effect of reducing labor pain and relieving maternal tension and anxiety, and there is no adverse reaction of mother and infant. This study analyzed the application value of multimodal analgesia (MMA) regimen of PCEA combined with auricular acupoint pressing, TENS, and acupoint injection in labor analgesia for primipara.

## 2. Materials and Methods

### 2.1. Research Object

A total of 300 singleton, full-term, head position primiparas, aged 20–30 years, at 37–42 weeks of gestation were selected from January to December 2021, all of them adopted natural delivery, all had no cephalopelvic disproportion or birth canal abnormalities, no obstetric or medical comorbidities, no immune system diseases, cardiovascular diseases, coagulation dysfunction, liver and kidney dysfunction, no contraindications to anesthesia, exclusion of placenta abruptio, placenta praevia, giant baby, and so on, all had normal communication ability, and the patient and family members had informed and signed consent. According to the different ways of labor analgesia, they were divided into the first stage of labor active period PCEA group (group A), the whole stage of labor PCEA group (group W), and the whole stage of labor PCEA combined with multiacupoint stimulation analgesia group (group WM). Comparing the general information in Table 1 for the three maternal groups, there were no statistical differences, and they were comparable (*P* > 0.05).

### 2.2. Inclusion Criteria

① Singleton, full-term, head position primiparas, aged 20–30 years, at 37–42 weeks of gestation were selected, and all of them adopted natural delivery. ② They were ASA class I-II. ③ They had no contraindications to vaginal delivery and anesthesia, no obstetric or medical comorbidities, no cephalopelvic disproportion or birth canal abnormalities, and so on. ④ They had no analgesic drugs or acupuncture points before entering labor and delivery and so on. ⑤ All had normal communication skills and signed consent forms for labor analgesia treatment.

### 2.3. Exclusion Criteria

The exclusion criteria included the following: ① multiple pregnancies, menstrual labor, weak contractions, intrauterine distress, fetal malposition, placenta abruptio, placenta praevia, and giant babies; ② contraindications of natural childbirth, transfer to cesarean section, pregnancy complications, and so on; ③ epidural block contraindications, skin damage or infection at the acupoint site, and so on; ④ severe organ dysfunction, mental and/or mental illness, and so on; ⑤ refusing labor analgesia and not signing the consent form for analgesia treatment.

### 2.4. Analgesic Regimen

Group A (the first stage of labor active period PCEA group): PCEA was performed when the first stage of labor active period (opening of the uterus to 3 cm) was reached. The puerpera was placed in the left lateral decubitus position with L2-3 epidural puncture and catheterization. After confirming that the catheter was located in the epidural space, 3 ml of 1% lidocaine was injected and observed for 5 minutes. If there were no adverse reactions, 10 ml of 0.1% ropivacaine combined with sufentanil 0.5 *μ*g/ml mixture was injected, and PCEA was performed 15 minutes later. The analgesic pump formula was 0.1% ropivacaine combined with sufentanil 0.5 *μ*g/ml, the background infusion rate was 5 ml/h, the additional volume was 6 ml, and the locking time was 15 min. PCEA was stopped at the end of the third stage of labor.

Group W (the whole stage of labor PCEA group): PCEA was performed when the first stage of labor incubation period was reached. The specific operation is the same as group A.

Group WM (the whole stage of labor PCEA combined with multiacupoint stimulation analgesia group): on the basis of group W, combined with multiacupoint stimulation analgesia during the whole-labor process, ① perform bilateral auricular pressure when entering the incubation period acupoints for the uterus, shenmen, internal genitalia, and sympathy were taken. The physician disinfected the auricle with alcohol, put the adhesive tape with vaccaria seed on the corresponding auricular points, pressed each point for 30 s/time, with the strength being appropriate to feel numbness, swelling, heat, acidity, and so on, pressed both auricular points alternately every 10 min, and stopped pressing the auricular points at the end of the first stage of labor; ② perform TENS when entering the incubation period, the main points were hegu and sanyinjiao, and the auxiliary points were zusanli. The Hua Tuo brand SDZ-II electronic needle therapy instrument (Suzhou Medical Supplies Co., Ltd.) was selected. The electrical stimulation frequency was 2 Hz, the wave width was 0.1 mA, the initial current intensity was 15 mA and gradually increased until the tremor was not painful, each treatment was 30 minutes, with an interval of 1 hour, and the two sides were alternately performed. TENS was stopped at the end of the third stage of labor; ③ perform acupoint injection when entering the incubation period, the ciliao and zhongliao were taken, the points were disinfected with iodophor, the puncture needle was pierced under the skin, and the needle was twisted and inserted; after getting acupuncture, 1 ml of 0.2% ropivacaine was injected into each point.

### 2.5. Observation Indicator

Labor pains: the visual analogue scale (VAS) was used to evaluate the analgesic effect of different analgesic regimens before analgesia (*T*_0_), at full opening of the uterus (*T*_1_), at the end of the second stage of labor (*T*_2_), and at the end of the third stage of labor (*T*_3_). The score ranged from 0 to 10; the higher the score, the more severe the degree.

Stress response: venous blood was collected to measure epinephrine (*E*), noradrenaline (NE), glucose (Glu), and *β*-endorphin (*β*-EP) levels at *T*_0_ and *T*_1_ in the three groups of mothers. All were measured by enzyme-linked immunosorbent assay, and the kits were from Dade Behring Inc.

Delivery time of each stage of labor: the delivery time of the first, second, and third stages of labor was compared among the three groups.

Physical condition of the newborns: at 1 and 5 minutes after birth, the Apgar score was used to evaluate the effect of different analgesic regimens on the physical condition of the newborns. The Apgar score included five items: activity, pulse, grimace, appearance, and respiration, each with a score of 0 to 2. The total score added up to 8–10 was considered normal, 4–7 was considered mild asphyxia, and <4 was considered severe asphyxia. The incidence of newborn asphyxia in the three groups was counted.

Indicators of umbilical artery blood gas analysis: umbilical artery blood was collected from the newborn immediately after delivery and transferred to the laboratory. A blood gas analyzer (ABL80, Radiometer Medical Equipment Co., Ltd.) was used to measure arterial blood PH value, base excess (BE), partial pressure of oxygen (PaO_2_), and partial pressure of carbon dioxide (PaCO_2_) in the three groups of newborns.

Postpartum depression (PPD): at 6 weeks after delivery, the Edinburgh PPD Scale (EPDS) was used to investigate the effect of different analgesia regimens on the occurrence of PPD.

### 2.6. Data Analysis

The data analysis software was SPSS 25.0, and the plotting software was GraphPad Prism 8.0. Measurement data were described by mean ± standard deviation, and the three groups were compared using a one-way analysis of variance and *t*-test for two-way comparisons. Count data were described by rate (%) and compared using the *χ*^2^ test. A two-sided test of *P* < 0.05 was considered as a statistically significant difference.

## 3. Results

### 3.1. Comparison of Analgesic Effects at Different Time Points in Three Groups of Mothers

At *T*_0_, there was no significant difference in the comparison of VAS scores among the three groups (*P* > 0.05). At *T*_1_, *T*_2_, and *T*_3_, the VAS scores were lower in groups W and WM than in group A, and the VAS scores were lower in group WM than in group W (*P* < 0.05), as indicated in Figure 1.

### 3.2. Comparison of Maternal Stress Responses in Three Groups at Different Time Points

At *T*_0_, there was no significant difference in the comparison of *E*, NE, Glu, and *β*-EP levels among the three groups (*P* > 0.05). At *T*_1_, the levels of *E*, NE, Glu, and *β*-EP were higher in the three groups than in the same group at *T*_0_, the levels of *E*, NE, and Glu were lower, the levels of *β*-EP were higher in groups W and WM than in group A, and the levels of *β*-EP were higher in group WM than in group W (*P* < 0.05), as indicated in Figure 2.

### 3.3. Comparison of the Delivery Time of Each Stage of Labor in Three Groups

Comparing the delivery time of the first stage of labor in the three groups, groups A and WM were shorter than group W (*P* < 0.05). Comparing the delivery time of the second and third stages of labor in all three groups, there was no significant difference (*P* > 0.05), as indicated in Figure 3.

### 3.4. Comparison of the Physical Condition in Three Groups of Newborns

Comparing the Apgar scores of the three groups of newborns at 1 and 5 min after birth, there was no significant difference (*P* > 0.05). Comparing the incidence of newborn asphyxia in the three groups, there was also no significant difference (*P* > 0.05), as indicated in Figure 4.

### 3.5. Comparison of Indicators of Umbilical Artery Blood Gas Analysis in Three Groups of Newborns

Comparing the PH, BE, PaO_2_, and PaCO_2_ of the three groups of newborns after delivery, there were no significant differences (*P* > 0.05), as indicated in Figure 5.

### 3.6. Comparison of the Incidence of PPD in Three Groups

At 6 weeks after delivery, the incidence of PPD was lower in groups W (10.00%) and WM (8.00%) than in group A (20.00%) (*P* < 0.05), as indicated in Figure 6.

## 4. Discussion

Normal physiological labor is mainly divided into the first, second, and third stages of labor. The nature of pain in each labor stage is different, which is mainly related to the differences in pain mechanism and innervation in different stages of labor [9]. To reduce maternal pain, in 2006, the American College of Obstetricians and Gynecologists advocated for a maternal request for pain relief as an indication for the administration of labor analgesia [10]. And more and more studies and guidelines believe that the implementation of epidural labor analgesia from the incubation period, that is, the implementation of epidural painless labor throughout the labor process, is safe and feasible [11].

Pain-induced stimuli can induce maternal stress, which can be suppressed by appropriate analgesia during labor [12]. *E* and NE are important indicators of the level of response to stress. When the body is stressed, the concentration of *E* and NE increases. If the mother is in a state of stress for a long time, it can cause immune and metabolic abnormalities [13, 14]. Glu is also an important indicator for evaluating maternal stress response. Under stress, the maternal release of catecholamines and glucocorticoids increases, insulin secretion is inhibited, glucagon release is accelerated, and ultimately Glu levels increase [15]. *β*-EP is an important opioid peptide in the human central nervous system that exerts analgesic effects by acting on the whole body [11]. According to the observation of this study, the VAS scores of the groups W and WM, which implemented incubation period PCEA, were lower than those of group A, which implemented active period PCEA, at *T*_1_, *T*_2_, and *T*_3_, and the VAS scores of group WM were lower than those of group W. At *T*_1_, the levels of *E*, NE, and Glu of groups W and WM were lower than those of group A, the levels of *β*-EP were higher than those of group A, and the levels of *β*-EP of group WM were higher than those of group W. It shows that the whole-labor MMA program reduces the levels of *E*, NE, and Glu, increases the level of *β*-EP, and relieves labor pain and stress response.

It is reported that although the pain in the latent period of the first stage of labor is not as obvious as in the active period, it still has physical and psychological effects on the mother [16]. In this study, the time of implementing analgesia in groups W and WM was earlier, which could reduce maternal psychological pressure and relieve physical pain earlier. And for multiacupoint stimulation and analgesia, auricular acupoints are selected according to the theory of meridians and the neurophysiological effects of auricular acupoints. Among them, shenmen acupoint can calm and relieve pain. Cooperating with the sympathetic point can effectively relieve the tension and anxiety of the puerperae and relieve the pain of childbirth. With the application of TENS, electroacupuncture at hegu can activate the endogenous analgesic system and promote the release of endogenous opioid *β*-EP to inhibit pain. Electroacupuncture at sanyinjiao can coordinate uterine contractions and relieve labor pain. Electroacupuncture at zusanli can reduce body stress and catecholamine levels to suppress labor pain. The application of acupoint injection, by injecting ropivacaine to ciliao and zhongliao points, can simultaneously close the spinal pain transmission gate and block the transmission of uterine pain information. Therefore, the whole-labor MMA of PCEA combined with multiacupoint stimulation for primipara can effectively reduce the pain of natural labor.

Pain during childbirth promotes the secretion of hormones such as *E* through nerve conduction and promotes uterine contraction and cervical dilation, thereby promoting the smooth progress of labor. However, excessive pain can cause adverse reactions such as electrolyte imbalance and cardiac load in puerperae, prolong the labor process, and affect the delivery outcome [17]. So, reasonable labor analgesia is very important. According to previous studies, latent period epidural analgesia can prolong the first stage of labor and increase the rate of cesarean section and the use of oxytocin. In the results of this study, there was no significant difference in the comparison of the second and third stage of labor delivery time among the three groups, and the first stage of labor time was shorter in groups A and WM than in group W, which is consistent with the above findings. Analyze the possible causes of the above results.” In this multiacupoint stimulation, pressure on the uterine points promotes uterine contractions. Cooperating with the internal genital point can accelerate the delivery of the fetus. Electroacupuncture at hegu can increase the intensity, frequency, and force of uterine contractions [18]. Electroacupuncture at sanyinjiao can excite the pelvic plexus and accelerate uterine contractions [19]. The multiacupoint stimulation effects cooperate with each other, thereby promoting the process of labor, shortening the time of labor, and increasing the rate of vaginal delivery.

While reducing the level of pain and stress during labor, labor analgesia also controls the level of elevated blood pressure and allows for a more adequate blood supply to the uterus, thus effectively reducing the risk of intrauterine distress in the fetus. The results of this study showed that there were no significant differences in the Apgar scores and umbilical artery blood gas analysis indices (PH, BE, PaO_2_, and PaCO_2_) between the three groups of newborns at 1 and 5 min after birth. It is suggested that the whole-labor MMA regimen has no adverse effects on the newborn and is safe. To analyze the reasons, the drugs ropivacaine and sufentanil used in PCEA in this study hardly pass the placental barrier, have no inhibition on neonatal breathing, and do not affect the uteroplacental blood circulation [20, 21]. And when it is combined with auricular acupoint pressing, TENS, and acupoint injection during the incubation period, it not only gives full play to the sedative and analgesic effects of multiple-acupoint stimulation to ensure full analgesia during labor but also fully ensures the safety of the newborn.

While most people think of pain during childbirth as a short-lived physiological event, for some women, persistent pain after childbirth can have a serious detrimental effect on their quality of life, whereas pain is directly associated with the development of depression, and the adverse effects of labor pain on mother and child are already present during the first stage of labor [22]. PPD is a series of depressive episodes of varying degrees that occur within 1 year after delivery and can adversely affect the intimate relationship between mother and child [23]. In the results of this study, at 6 weeks postpartum, the incidence of PPD in group W (10.00%) and group WM (8.00%) was lower than that in group A (20.00%). It indicates that good labor analgesia during the whole stage of labor can better reduce the pain and anxiety caused by labor pain, thereby reducing the occurrence of PPD.

The shortcoming of this study is that the relationship between labor analgesia and PPD has not been studied in the long term, considering the inconvenience of long-term postoperative follow-up or the problems of missed visits. It is generally accepted that puerperal depression is diagnosed if EPDS scores ≥13 at 6 weeks postpartum [24]. The observation period of this study was short, and the observation of the long-term effects of full labor multimodal labor analgesia with multiple-acupoint stimulation on PPD in primiparas remains to be further studied in the future.

## 5. Conclusion

The application of the MMA regimen of PCEA combined with multiacupoint stimulation for labor analgesia during the whole stage of labor in primipara can effectively reduce labor pain and stress response during the whole stage of labor and shorten the delivery time of the first stage of labor, the indicators of newborn Apgar score and umbilical artery blood gas analysis are not affected, and the incidence of PPD in patients is reduced, which can play a protective role for the safety of mother and infant.

## Figures and Tables

**Figure 1:** Comparison of analgesic effects at different time points in the three groups of mothers. *Note.*^*∗*^indicates *P* < 0.05 compared with simultaneous points in group A; ^#^indicates *P* < 0.05 compared with simultaneous points in group W.

**Figure 2:** Comparison of maternal stress responses in the three groups at different time points. (a) E levels at *T*0 and *T*1 in three maternal groups. (b) NE levels at *T*0 and *T*1 in three maternal groups. (c) Glu levels at *T*0 and *T*1 in three maternal groups. (d) *β*-EP levels at *T*0 and *T*1 in three maternal groups. ^*∗*^indicates *P* < 0.05 compared with the same group at *T*0; ^#^indicates *P* < 0.05 compared with group A at *T*1; ^^^ indicates *P* < 0.05 compared with group W at *T*1.

**Figure 3:** Comparison of the delivery time of each stage of labor in the three groups. *Note.*^*∗*^indicates *P* < 0.05 compared with the first stage of labor in group W.

**Figure 4:** Comparison of the physical condition of the three groups of newborns. (a) Apgar scores of newborns in the three groups. (b) Incidence of newborns asphyxia in the three groups.

**Figure 5:** Comparison of indicators of umbilical artery blood gas analysis in the three groups of newborns. (a) PH in the three groups of newborns. (b) BE in the three groups of newborns. (c) PaO2 in the three groups of newborns. (d) PaCO2 in the three groups of newborns.

**Figure 6:** Comparison of the incidence of PPD in the three groups. *Note.*^*∗*^indicates *P* < 0.05 compared with group A.

**Table 1:** General information of the three maternal groups.

Group	n	Age (years)	Gestational weeks (weeks)	Height (cm)	Weight (kg)
Group A	100	25.88 ± 1.60	39.35 ± 0.67	160.33 ± 2.29	65.85 ± 2.11
Group W	100	25.42 ± 1.54	39.32 ± 0.69	160.22 ± 2.27	65.96 ± 2.04
Group WM	100	25.77 ± 1.46	39.35 ± 0.67	160.26 ± 2.30	65.93 ± 2.20
*F*		2.451	0.066	0.593	0.072
*P*		0.088	0.937	0.942	0.932

## Data Availability

The data analyzed or used in the current study are available from the corresponding author.
